The article "Coral-Bacterial Communities before and after a Coral Mass Spawning Event on Ningaloo Reef" was published in 2012. Journal: PLoS One.

# Coral-Bacterial Communities before and after a Coral Mass Spawning Event on Ningaloo Reef

**DOI:** 10.1371/journal.pone.0036920

**Published:** 2012-05-16

**Authors:** Janja Ceh, Jean-Baptiste Raina, Rochelle M. Soo, Mike van Keulen, David G. Bourne

**Affiliations:** 1 School of Biological Sciences and Biotechnology, Murdoch University, Perth, Western Australia, Australia; 2 Centre for Marine Microbiology and Genetics Research, Australian Institute of Marine Science, Townsville, Queensland, Australia; 3 , ARC Centre of Excellence for Coral Reef Studies, and School of Marine and Tropical Biology, James Cook University, Townsville, Queensland, Australia 3AIMS@JCU; Leibniz Center for Tropical Marine Ecology, Germany

## Abstract

Bacteria associated with three coral species, *Acropora tenuis*, *Pocillopora damicornis* and *Tubastrea faulkneri*, were assessed before and after coral mass spawning on Ningaloo Reef in Western Australia. Two colonies of each species were sampled before and after the mass spawning event and two additional samples were collected for *P. damicornis* after planulation. A variable 470 bp region of the 16 S rRNA gene was selected for pyrosequencing to provide an understanding of potential variations in coral-associated bacterial diversity and community structure. Bacterial diversity increased for all coral species after spawning as assessed by Chao1 diversity indicators. Minimal changes in community structure were observed at the class level and data at the taxonomical level of genus incorporated into a PCA analysis indicated that despite bacterial diversity increasing after spawning, coral-associated community structure did not shift greatly with samples grouped according to species. However, interesting changes could be detected from the dataset; for example, *α-Proteobacteria* increased in relative abundance after coral spawning and particularly the *Roseobacter* clade was found to be prominent in all coral species, indicating that this group may be important in coral reproduction.

## Introduction

Corals exhibit a range of reproductive strategies, which include both sexual and asexual propagation. Brooding coral species show internal fertilization and expel well-developed larvae at various times of the year, usually over the summer months. Most corals however reproduce during annual spawning events, by broadcast spawning their gametes for external fertilisation [1]. Mass spawning is a well known phenomenon occurring worldwide and involves the synchronous release of gametes from benthic invertebrates including scleractinian corals. The timing of coral mass spawning depends on the geographical location, and usually occurs in summer, once a year over a few nights following the full moon [1]. Coral reproduction is regulated by several life processes such as gamete production, fertilization, planktonic larval dispersal, larval settlement, post-settlement growth, and survival. Disruption in these early life stages can result in compromised or failed recruitment and profoundly affect the distribution and survival of corals [2].

The article "Coral-Bacterial Communities before and after a Coral Mass Spawning Event on Ningaloo Reef" was published in 2012. Journal: PLoS One.

A stimulation of microbial processes within reef waters after episodic spawning events has previously been reported [3], [4]. After a coral mass spawning event on the Great Barrier Reef (GBR), bacterial abundances in reef water increased 2-fold and remained elevated for three days, before declining to below pre-spawning values [4]. The input of large quantities of particulate organic matter in the form of degrading gametes enhance pelagic and benthic autotrophic and heterotrophic activities [5], and can result in rapid oxygen depletion in the water column [6].

Microbes in coral reef ecosystems have been extensively studied with regard to their role in coral health and disease [7], coral antimicrobial properties [8] and their involvement in the biogeochemical cycling of nutrients [9], [10]. Furthermore microbes have been suggested to co-evolve with their coral host [7] and to benefit the coral in adapting to environmental changes in the ecosystem [11]. Previous studies suggested that bacterial communities in corals are distinct from those inhabiting the surrounding seawater [12] and that some corals harbour specific bacteria species, despite temporal or geographical separation [13], [14]. Conversely, other studies showed that bacterial consortia varied with location [15] and time [16], indicating that coral–microbial community structures may be either a result of environmental drivers [16], [17] or species- and site specific [18]. Understanding the acquisition, maintenance and successional changes of microbial communities through different coral life stages is fundamental to understanding the functional roles these partnerships have in overall coral health.

Energy demanding physiological processes such as reproduction affect the corals metabolism which may impact its numerous microscopic partners (including *Symbiodinium*, Bacteria, Archaea, Fungi and viruses which form a functionally relevant mutualistic relationship with coral known as the coral holobiont) [14]. Coral reproduction itself as well as the environmental changes associated with the large scale ecological event of coral mass spawning could potentially influence coral bacterial associates. If corals acquire bacteria according to their specific requirements in different life stages, reproduction accomplished colonies might rid themselves of bacteria associated with and important to reproduction and recruit alternative bacteria populations more suitable for the time after spawning. Coral bacteria might also change due to corals releasing large quantities of beneficial bacteria with their gametes (spawners) or planula larvae (brooders), and the re-colonization with new bacteria; or corals may simply return to pre-spawning bacterial populations as observed for temperature stressed and bleached corals [19].

The article "Coral-Bacterial Communities before and after a Coral Mass Spawning Event on Ningaloo Reef" was published in 2012. Journal: PLoS One.

This study investigated the diversity and community structure of coral-associated bacterial communities before and after a coral mass spawning event. Three coral species were assessed: the broadcast spawning coral *A. tenuis* (which participated in the synchronous event), the brooding coral *P. damicornis* (additional samples were collected for this species after its respective reproductive event), and the ahermatypic coral *T. faulkneri*. *T. faulkneri* does not associate with the algal symbiotic partner *Symbiodinium* which has previously been suggested to be involved in structuring coral microbial communities [20], [21]. Like *P. damicornis*, the ahermatypic coral *T. faulkneri* broods and releases planulae and was intended to serve as an ahermatypic example. However no reproductive activity was observed through the study time (one month of observation) and the timing of reproduction for this species is unknown for the Ningaloo Reef system. Bacterial diversity was assessed by a 16 S rRNA gene pyrosequencing approach allowing for large-scale exploration of taxonomic diversity. This study is the first to investigate the dynamics of coral-microbial associates before and after coral reproductive stages.

## Methods

### Sample Site and Sample Collection

Three coral species, *P. damicornis*, *A. tenuis* and *T. faulkneri* were used in this study. Two replicated colonies per coral species were tagged and sampled on a reef flat (5–6 m water depth) near Coral Bay (23° 07′S, 113° 07′E), Ningaloo Reef, Western Australia. For each species, two pieces were collected (one from each replicate colony) two days before and two days after the coral mass spawning event in March 2009. Two additional *P. damicornis* colonies were removed from the reef structure and kept in an open plastic container (80×50×50 cm) on the reef flat during the day and assessed for reproductive activity on the beach at night time. The container was kept in knee deep water to maintain the ambient water temperature and returned to the reef at sunrise. *P. damicornis* released their planulae one week after the mass spawning event and were sampled on the reef two days after the last reproductive activity.

The article "Coral-Bacterial Communities before and after a Coral Mass Spawning Event on Ningaloo Reef" was published in 2012. Journal: PLoS One.

Two similar sized coral nubbins (approximately 2 cm in size) were removed from two coral colonies of each species using a bone clipper. Coral nubbins were placed immediately into individual, sterile zip-lock plastic bags under water and rinsed 3 times with artificial seawater (0.2 µm filtered and autoclaved) on the surface and placed on ice. The coral samples were air brushed with 2 ml of ASW to remove the coral tissue including the associated microorganisms from the coral skeleton and the tissue slurry aliquoted into cryovials. All samples were stored at −80°C until required for analysis. Samples were processed within one hour of sampling. Permits for this study were provided by the Department of Environment and Conservation.

### DNA Extraction and PCR and Sequencing Preparation

Frozen tissue samples from all sampled corals were aseptically transferred to 1.5 ml Eppendorf tubes and total genomic DNA extracted using the MO BIO PowerPlant DNA Isolation Kit as per the manufacturer’s instructions (MO BIO Laboratories, CA, USA). Extracted DNA was quantified using a GeneQuant Pro spectrophotometer (Amersham Pharmacia Biotech) and stored at –20°C until required.

A 470 bp region of the 16 S ribosomal RNA gene (16 S rRNA) including the variable regions 1–3 was selected for tag pyrosequencing using the bacterial forward primer 63 F which included the primer A adaptor on the 5′ end along with a unique 8 bp barcode (5′- CCATCTCATCCCTGCGTGTCTCCGACTCAGNNNNNNNNCAGGCCTAACACATGCAAGTC) and the bacterial reverse primer 533 R with the primer B adaptor on the 5′end (5′- CCTATCCCCTGTGTGCCTTGGCAGTCTCAGTTACCGCGGCTGCTGGCAC). All amplifications were run under the following conditions: 1×Qiagen PCR Buffer (Qiagen, Germany), 1 U of HotStarTaq DNA Polymerase (Qiagen), 200 µM of each deoxynucleotide triphosphate (dNTP), 25 pmoles of each primer and MilliQ water up to 50 µl. Equal volumes of DNA (20 ng total) from each sample were used as template to generate PCR amplicons (tags). Thermocycling conditions for the amplification consisted of an initial ‘enzyme activation’ at 95°C for 5 min, followed by 30 cycles of 94°C for 1 min, 55°C for 1 min and 72°C for 1 min, followed by a final extension step of 72°C for 10 min. A total of 5 PCRs were performed for each sample and the replicate PCR’s pooled to generate more than 1 µg of template DNA. PCR products were purified using the MO Bio PCR purification kit as per the manufacturer’s instructions. Note: three of the *P.* damicornis (before, after spawning and after planulation) and one of the *T. faulkneri* samples (after spawning) failed to amplify and were excluded from subsequent analysis. The amount of DNA in each sample was quantified using the Quant-iT PicoGreen assay (Invitrogen, Carlsbad, CA). All samples with their respective bar codes (10 samples in total) were pooled in equimolar amounts for 454 pyrosequencing on a Roche GS-FLX system at the Australian Genome Research Facility (AGRF) Brisbane, Australia.

The article "Coral-Bacterial Communities before and after a Coral Mass Spawning Event on Ningaloo Reef" was published in 2012. Journal: PLoS One.

### Sequence and Statistical Analyses

The sequence fasta and quality files were extracted from the raw sff output from the 454 sequence run and the sequence tag and its associated quality scores were removed. The python script split_libraries.py from the QIIME pipeline [22] was used to remove poor quality (<25) and short sequences (<150 bp), remove the primer and barcode, and add a sample identifier to the header of each sequence. The resulting fasta file was checked for chimeric sequences against a chimera-free database of 16 S rRNA gene sequences (Green Genes 29/11/10 release) using UCHIME [23]. All sequences that were identified as potential chimeras were removed. Homopolymer sequence errors were corrected using ACACIA (pers.com. Dr. Gene Tyson) resulting in a chimera and error-free fasta file. The number of reads per sample was quantified for each of the previous steps (see Table 1). The number of chimera-free and error-free reads was normalised to 475 reads per sample to allow comparative diversity analysis between all samples. No significant differences (P = 0.01; 1000 permutations) were observed between the raw, cleaned and normalised datasets when PCA analysis was performed on the relative abundance of the dominant OTUs and correlation between datasets was assessed by Procrustes rotation [24]. Therefore all analysis reported in this study was conducted on the randomly subsampled and normalised dataset. Sequences were clustered using uclust [25] to obtain groups of sequences at both the 90% and 97% similarity levels. These groups represent operational taxonomic units (OTUs) defined at an approximate ‘genus’ and ‘species’ levels. The QIIME pipeline was used to identify the most abundant member of each group which was subsequently chosen as the representative sequence. Sequence taxonomy was assigned using GreenGenes [26] and BLAST (0.75 similarity) and the QIIME pipeline was used to generate OTU tables. Alpha diversity statistics in QIIME were calculated after random sub-sampling to ensure sequencing effort did not affect diversity comparisons. Once the data set was rarefied, the following alpha-diversity metrics were generated; total observed species (OTUs) and Chao 1 diversity. Beta-diversity of the bacterial communities was analysed in using weighted UNIfrac analysis with principal components generated from the UniFrac distances and plotted in two dimensions. The pyrosequencing dataset were deposited in the NCBI Sequence Read Archive (SRA) database with the accession number (pending).

The article "Coral-Bacterial Communities before and after a Coral Mass Spawning Event on Ningaloo Reef" was published in 2012. Journal: PLoS One.

**Table 1:** Sampling times and statistical diversity parameters.

Samples/Species	*A. tenuis* *(1)*	*A. tenuis* *(2)*	*P. damicornis* *(1)*	*T. faulkneri* *(1)*	*T. faulkneri* *(2)*	*A. tenuis* *(1)*	*A. tenuis* *(2)*	*P. damicornis* *(1)*	P. damicornis* *(1)*	*T. faulkneri* *(1)*
Sampling time	before coral mass spawning					after coral mass spawning				
High quality seqs.	932	1031	595	1598	1247	2008	1566	492	475	1966
Rarified seqs.	475	475	475	475	475	475	475	475	475	475
OTU_0.03_	140	181	54	359	222	357	272	63	127	473
Chao 1_0.03_	148.606	208.991	71.038	377.421	220.389	412.396	269.426	111.446	242.625	503.815

An analysis of similarities (ANOSIM) was performed to compare bacterial species diversity between coral species. A test run on R, using the package “vegan” identified significant differences in bacterial communities between coral species; the significance was computed by the permutation of the group membership, with 10,000 replicates and Bray-Curtis distance as a distance measure.

## Results

Samples collected from *A. tenuis*, *P. damicornis* and *T. faulkneri* before and after coral mass spawning and after planulation for *P. damicornis* provided a total of 11910 high quality 16 S rRNA gene sequence tags (Table 1). Chao 1 diversity index revealed the highest and lowest diversity of bacteria in *T. faulkneri* and *P. damicornis*, respectively. Bacterial diversity increased in all coral species after coral spawning, additionally bacterial diversity increased after planulae release in *P. damicornis.*

Replicate samples were highly similar for each time point (with the exception of the *γ-Proteobacteria, Pseudoalteromonas* and *Shigella*, which varied in their abundance between replicates in *A. tenuis* samples), they were therefore pooled for clarity purposes. Pooled sequence libraries provided a general overview over the ten most abundant bacteria classes associated with coral samples (Fig. 1). The *γ-Proteobacteria* was the dominant class of bacterial associated with all the corals. *α-Proteobacteria* retrieved sequences were also consistently retrieved from all the coral samples. *Bacilli* were consistently found in the *P. damicornis* corals while the *Flavobacteria* were consistently present in *A. tenuis* and *T. faulkneri* samples. No major shifts in coral bacterial communities were observed at the class level before and after the coral mass spawning event. This observation was consistent for all coral species and any detected variations were only minor changes in abundance of bacterial classes. *A. tenuis* and *P. damicornis* displayed more similar bacteria classes whereas sequence libraries derived from the ahermatypic coral *T. faulkneri* differed from the other two coral species. Coral samples grouped according to species at the class level (Fig. 1).

The article "Coral-Bacterial Communities before and after a Coral Mass Spawning Event on Ningaloo Reef" was published in 2012. Journal: PLoS One.

**Figure 1:** Bacterial 16 S rRNA gene sequences retrieved from three coral species before (b), after (a) coral spawning and after planulation (a*). Replicate samples were pooled and dominant affiliations were grouped at the class level. The similarity tree was done using the neighbour-joining method and the Bray-Curtis algorithm (n = 1000 replications). Note: due to failure in amplification *P. damicornis* and *T. faulkneri* are represented by one sample per sampling point and one sample after coral spawning, respectively.

A principal component analysis (PCA) of the individual sequence data sets (unpooled samples) based on a taxonomic assignment at the genus level (>97% identity for OTU groupings) again revealed that all samples grouped according to coral species (Fig. 2) and all coral species displayed significantly different bacterial communities between each other (R = 1, rb = 6.5, rw = 35, p<0.0003). Coral replicates collected after coral spawning displayed some shifts in the coral microbial community structure when compared with samples collected directly before spawning. Furthermore slight variations in coral microbial assemblages were amplified for *P. damicornis* after planulation.

**Figure 2:** Principal component analysis (PCA) of 16 S rRNA gene sequences, showing non-pooled coral samples grouped into OTUs>97% identity, before, after coral spawning and after planulation.

Sequence tags grouped into OTUs at >97% identity were considered dominant in any sample collected when present at proportions of >1%. This resulted in the 35 most abundant out of a total number of 116 OTUs, covering 92% of all retrieved sequences (Table 2). Sequence affiliations included the classes of *Acidobacteria*, *Flavobacteria*, *Sphingobacteria, Bacilli, Clostridia, α-, β- and γ-Proteobacteria* (Table 2). Six of 35 OTUs were present in all coral species out of which only two were found at all collection times (Table 2). *A. tenuis* samples consisted of 20, *P. damicornis* of 14 and *T. faulkneri* of 24 of the most abundant OTUs.

Only seventeen percent of the most abundant OTUs (five percent of all OTUs) were shared between all coral species investigated, and were associated with the *α-Proteobacteria Rhodomicrobium, Roseobacter*, and *Rhodospirillales* and the *γ-Proteobacteria Shewanella, Pseudoalteromonas* and *Stenotrophomonas* (Fig. 3).

**Table 2:** OTU’s (grouped at 97% identity) of the most abundant bacteria from three coral species before (b), after (a) coral spawning and after planulation (a*); sequences of proportions >1% were included and numbers represent percentages of sequence affiliations.

OTU’s	*A. tenuis*		*P. damicornis*			*T. faulkneri*	
	b	a	b	a	a*	b	a
***Bacteria; Acidobacteria; Acidobacteria; Acidobacteriales; Acidobacteriaceae,*** ** unclassified**	14	7			3		
***Bacteria; Bacteroidetes; Flavobacteria; Flavobacteriales,*** ** unclassified, unclassified**							1
***Bacteria; Bacteroidetes; Flavobacteria; Flavobacteriales; Flavobacteriaceae,*** ** unclassified**	4	7				4	4
***Bacteria; Bacteroidetes; Flavobacteria; Flavobacteriales; Flavobacteriaceae; Tenacibaculum***						2	
***Bacteria; Bacteroidetes; Sphingobacteria; Sphingobacteriales,*** ** unclassified, unclassified**							2
***Bacteria; Bacteroidetes; Sphingobacteria; Sphingobacteriales; Flexibacteraceae, unclassified***							3
***Bacteria; Firmicutes; Bacilli; Bacillales; Bacillaceae; Bacillaceae 1***			45	16	7		
***Bacteria; Firmicutes; Clostridia; Clostridiales; Incertae Sedis XII, unclassified***					2		
***Bacteria; Firmicutes; Clostridia; Clostridiales; Incertae Sedis XII; Fusibacter***					5		
***Bacteria; Proteobacteria; α-Proteobacteria; Rhizobiales,*** ** unclassified, unclassified**		1					
***Bacteria; Proteobacteria; α-Proteobacteria; Rhizobiales; Hyphomicrobiaceae; Rhodomicrobium***	2	2	1	1	6	3	2
***Bacteria; Proteobacteria; α-Proteobacteria; Rhodobacterales; Rhodobacteraceae, Roseobacter***	6	8			5	12	13
***Bacteria; Proteobacteria; α-Proteobacteria; Rhodobacterales; Rhodobacteraceae; Silicibacter***		1				3	1
***Bacteria; Proteobacteria; α-Proteobacteria, Rhodospirillales,*** ** unclassified, unclassified**	3	4			2	4	3
***Bacteria; Proteobacteria; α-Proteobacteria; Sphingomonadales; Sphingomonadaceae; Erythrobacter***	10	18				1	2
***Bacteria; Proteobacteria; α-Proteobacteria; Sphingomonadales; Sphingomonadaceae; Novosphingobium***			2	1	2		
***Bacteria; Proteobacteria; α-Proteobacteria; Sphingomonadales; Sphingomonadaceae; Sphingomonas***		1					
***Bacteria; Proteobacteria; γ-Proteobacteria; Alteromonadales,*** ** unclassified, unclassified**	4	5				6	8
***Bacteria; Proteobacteria; γ-Proteobacteria; Alteromonadales; Alteromonadaceae,*** ** unclassified**		1				1	3
***Bacteria; Proteobacteria; γ-Proteobacteria; Alteromonadales; Alteromonadaceae; Aestuariibacter***	4	4				2	4
***Bacteria; Proteobacteria; γ-Proteobacteria; Alteromonadales; Alteromonadaceae; Alteromonas***		2					4
***Bacteria; Proteobacteria; γ-Proteobacteria; Alteromonadales; Colwelliaceae,*** ** unclassified**						1	1
***Bacteria; Proteobacteria; γ-Proteobacteria; Alteromonadales; Colwelliaceae; Thalassomonas***						6	2
***Bacteria; Proteobacteria; γ-Proteobacteria; Alteromonadales; Incertae sedis 7,*** ** unclassified**						2	4
***Bacteria; Proteobacteria; γ-Proteobacteria, Alteromonodales; Shewanellaceae, Shewanella***	7	6	1	2	11	16	13
***Bacteria; Proteobacteria; γ-Proteobacteria; Alteromonadales; Pseudoalteromonadaceae; Pseudoalteromonas***	2	7	2	1		21	2
***Bacteria; Proteobacteria; γ-Proteobacteria; Enterobacteriales; Enterobacteriaceae,*** ** unclassified**	2						
***Bacteria; Proteobacteria; γ-Proteobacteria; Enterobacteriales; Enterobacteriaceae; Shigella***	22	10					
***Bacteria; Proteobacteria; γ-Proteobacteria; Oceanospirillales; Oceanospirillaceae,*** ** unclassified**					3		2
***Bacteria; Proteobacteria; γ-Proteobacteria; Oceanospirillales, Oceanospirillaceae, Oceanospirillum***					1		16
***Bacteria; Proteobacteria; γ-Proteobacteria; Pseudomonadales; Moraxellaceae; Acinetobacter***			33	53	27	4	
***Bacteria; Proteobacteria; γ-Proteobacteria; Vibrionales; Vibrionaceae,*** ** unclassified**	1						
***Bacteria; Proteobacteria; γ-Proteobacteria; Vibrionales; Vibrionaceae; Vibrio***	7	2					
***Bacteria; Proteobacteria; γ-Proteobacteria; Xanthomonadales; Xanthomonadaceae; Stenotrophomonas***		1	9	18	16	4	
**Unclassified Bacteria**	4	4				1	2

The article "Coral-Bacterial Communities before and after a Coral Mass Spawning Event on Ningaloo Reef" was published in 2012. Journal: PLoS One.

**Figure 3:** Variation in OTUs representing bacterial groups that are potentially important in coral reproduction.

## Discussion

Three coral species, *A. tenuis*, *P. damicornis* and *T. faulkneri* were examined to explore shifts in coral associated bacterial assemblages before and after a coral mass spawning event. Bacterial diversity increased after reproductive activity for both coral species, *A. tenuis* after coral spawning and *P. damicornis* after planulation, as indicated by Chao 1 index.

No major shifts in coral bacterial communities were observed at the class level through the coral reproduction event. This observation was consistent for all coral species which demonstrated similar microbial communities with only minor variations in abundances between bacterial classes. A more precise taxonomical assignment at the genus level (97% similarity) indicated similarities between *A. tenuis* and *T. faulkneri* in both, proportions and identities of their bacterial communities. *P. damicornis* however displayed differences in bacterial composition compared to the other two coral species. Only seventeen percent of the most abundant OTUs were shared between all coral species investigated, and were associated with the *α-Proteobacteria Rhodomicrobium, Roseobacter*, and *Rhodospirillales* and the *γ-Proteobacteria Shewanella, Pseudoalteromonas* and *Stenotrophomonas* Corals have previously been reported to harbour specific bacteria which differ from bacterial communities in the seawater [12] and the aforementioned bacteria groups seem to represent a consistent and important component in coral-bacterial associations with *A. tenuis*, *P. damicornis* and *T. faulkneri*, whereas other bacterial groups not found to be consistently dominant are likely to vary between coral species.

The article "Coral-Bacterial Communities before and after a Coral Mass Spawning Event on Ningaloo Reef" was published in 2012. Journal: PLoS One.

Investigating the taxonomic assignment at the genus level revealed a specific partition for bacterial classes associated with corals. For example within the family *Sphingomonadaceae*, the genus *Erythrobacter* was present in *A. tenuis* and in *T. faulkneri* only, whereas *Novosphingobium* was only represented in *P. damicornis*. Increased retrieval of sequences related to the genera *Erythrobacter* and *Pseudoalteromonas* potentially highlight their significance in *A. tenuis* reproduction; both genera are commonly known to associate with corals [13], [14], [27] and can inhibit the growth of the coral pathogen *Vibrio coralliilyticus* [28]. Furthermore, *Pseudoalteromonas* has previously been shown to induce coral settlement [29] and to possess antimicrobial properties [8], [30].

Interestingly all bacteria types affiliated with the class *α-Proteobacteria* either increased or remained unchanged in relative proportion of retrieved sequences after reproduction in the corals *A. tenuis* and *P. damicornis* compared to pre-spawning samples. This suggests that *α-Proteobacteria* may be important in coral reproduction including possible implications for the survival and increase of fitness in coral larvae. Previous work reported the genus *Roseobacter* to be amongst the first acquired bacteria in early developing stages of the coral *Pocillopora meandrina* [31], [32]. *Roseobacter* clade affiliated bacteria species are abundant and diverse in seawater and various metabolic functions have been reported for this taxon [33], including antibiotic properties against coral pathogens [34]. In the present study *Roseobacter* affiliated sequences are prominent in all coral species and represent the only bacteria type increasing after spawning as well as after planulation (Fig. 3), possibly providing antimicrobial activity against potentially pathogenic bacteria for coral compromised after energy demanding life stages such as spawning [35]. These findings support the idea that *Roseobacter* affiliated bacteria may be specifically related to the process of reproduction in brooding as well as in spawning corals.

This is the first study to directly compare shifts in coral bacterial associations before and after spawning. Coral species displayed similar classes of bacteria, though at the genus level, small differences in associated bacterial communities were observed. Abundant OTUs potentially represent bacteria which play a role during coral reproduction since they specifically appeared before or after coral spawning or in distinctly high numbers in between sampling times. This study lays the groundwork for future research investigating potentially important functional roles of the identified bacterial groups, and their implication in coral reproduction and the early establishment of corals.
